The article "Cryptotanshinone Protects against PCOS-Induced Damage of Ovarian Tissue via Regulating Oxidative Stress, Mitochondrial Membrane Potential, Inflammation, and Apoptosis via Regulating Ferroptosis" was retracted in 2023. Reasons: signs of a paper mill; suspected computer-generated content; unreliable results or conclusions; concerns about the data.

# Cryptotanshinone Protects against PCOS-Induced Damage of Ovarian Tissue via Regulating Oxidative Stress, Mitochondrial Membrane Potential, Inflammation, and Apoptosis via Regulating Ferroptosis

**DOI:** 10.1155/2022/8011850

**Published:** 2022-04-04

**Authors:** Honglin Liu, Jiani Xie, Limin Fan, Yue Xia, Xia Peng, Jianhua Zhou, Xiaorong Ni

**Affiliations:** ^1^Department of Gynecology, Shanghai University of Traditional Chinese Medicine, Shanghai Traditional Chinese Medicine Hospital, 274 Middle Zhi Jiang Rd, Shanghai 200071, China; ^2^The Institute for Biomedical Engineering and Nano Science Tongji University School of Medicine, No. 1239, Siping Road, Shanghai 200092, China

## Abstract

Polycystic ovary syndrome (PCOS) is the most common endocrine disorder in women of childbearing age. Cryptotanshinone (CRY) has been shown to be effective in reversing reproductive disorders, but whether it can be used in the treatment of polycystic ovary syndrome remains unclear. We aimed to explore whether the mechanism of cryptotanshinone (CRY) in the treatment of polycystic ovary syndrome (PCOS) can be driven via regulating ferroptosis. A rat model of PCOS was established by daily injection of human chorionic gonadotropin and insulin for 22 days. An in vitro model of ischemia-reperfusion (IR) of granulosa cells was established. The in vitro and rat models of PCOS were subjected to different treatments including ferroptosis activators and inhibitors, CRY, and MAPK inhibitor. Oxidative stress was evaluated by measuring the activities of SOD, MDA, and GSH-PX. Total body weight and ovarian weight, as well as the levels of LH and the LH to FSH ratio, significantly increased in rats with PCOS, compared with controls. The expression of Bax was increased in PCOS tissues while PGC1*α*, NFR1, GPX4, catalase p-ERK, and Bcl-2 were all downregulated. Ferroptosis activator, erastin, had effects similar to those of PCOS while the contrary was found with CRY and ferroptosis inhibitor treatment groups. In vitro, CRY inhibited oxidative stress, MMP, and NF-*κ*B and activated MAPK/ERK signaling by regulating ferroptosis. Overall, this study indicated that CRY protects against PCOS-induced damage of the ovarian tissue, via regulating oxidative stress, MMP, inflammation, and apoptosis via regulating ferroptosis.

## 1. Introduction

Polycystic ovary syndrome is an endocrine disease affecting 15%-20% of women of childbearing age [1]. The etiology and pathogenesis of PCOS are unknown, and the diagnosis is often delayed. The repercussions of PCOS are varied and include psychological, gynecological, and metabolic disorders such as insulin resistance, type II diabetes, cardiovascular risks, and obesity; PCOS is also one of the causes of infertility in women due to the ovulatory disorders it triggers [2–6]. To date, there is no effective treatment to cure PCOS and the proposed treatments are symptomatic and are aimed at correcting the symptoms related to hyperandrogenism, restoring the menstrual cycle to increase the chances of fertility, and correcting metabolic abnormalities [7–9]. For PCOS patients with infertility, infertility treatment options such as drugs (letrozole, clomiphene citrate, and gonadotropins), surgery, and in vitro fertilization are offered to patients [10, 11]. Therefore, given the urgency of the situation, it is necessary to look for ways to develop effective treatments for PCOS.

Cryptotanshinone is one of the major bioactive molecules extracted from the plant Salvia miltiorrhiza Bunge (Danshen), a plant recognized in traditional Chinese medicine for its virtues in the treatment of various diseases [12]. Previous studies have shown that CRY has biological activities for the treatment of diseases such as coronary heart disease, kidney failure, Alzheimer's disease, cancers, obesity, ageing, diabetes, and fibrosis of the liver, lungs, heart, and kidneys [13–23]. A limited amount of research has shown that CRY may be effective in the treatment of PCOS and some molecular mechanisms have been proposed [24–27]. In our previous study [28], we also demonstrated the efficacy of CRY in the treatment of PCOS and proposed that its mode of action is mediated by its effect on the regulation of the HMGB1/TLR4/NF-kappaB signaling pathway. However, given the complexity of the pathogenesis and pathophysiology of PCOS, it is important to further investigate the molecular mechanisms underlying PCOS and to explore the mechanisms of action of CRY in order to propel this molecule in the treatment of PCOS.

Ferroptosis is a type of necrotic cell death that has been implicated in the pathogenesis of various diseases such as cancers, cardiovascular diseases, neurodegenerative diseases, diabetes, and renal failure [29–36]. Studies have shown that ferroptosis is at the center of a multitude of metabolic pathways [31, 33], which gives it a key role in understanding and developing therapeutics. Indeed, studies have demonstrated an interconnection between ferroptosis and biological processes such as oxidative stress and mitochondrial function [37–39]. The current trend suggests that modulation of ferroptosis, either through its inhibition or activation, could be beneficial for the treatment of many diseases. However, although few studies have suggested the involvement of ferroptosis in processes related to ovarian disorders, the role of ferroptosis in PCOS remains unknown. In addition, it has been reported that cryptotanshinone against lung cancer cells is through ferroptosis [40]. Also, cryptotanshinone may increase the accumulation of ROS by inhibiting the expression of xCT and GPX4 to induce the ferroptosis of HepG2 cells [41]. Furthermore, despite the potential of CRY in the treatment of various diseases, no published study, to the best of our knowledge, has yet scrupulously analyzed whether ferroptosis could be a target of the mechanism of action of CRY in the treatment of PCOS or other diseases. Thus, the novelty and motivation of this study are to expand our knowledge on the mechanisms of action of CRY and its impact on ferroptosis in PCOS would be of great importance in the treatment of PCOS and various diseases.

Thus, in the present study, we set out to extend our previous research by exploring the effect of CRY on ferroptosis and related biological processes such as oxidative stress and mitochondrial function.

## 2. Material and Methods

### 2.1. The Rats Used in the Experiments

The rats used in this study were commercially acquired from the Shanghai Laboratory Animal Center, Co. Ltd. The weight of the rats was in the range of 174-210 g, and their average age was 87.8 days. The rats were housed and acclimatized in a temperature-controlled environment of 25 ± 2°C with alternating cycles of 12 h of darkness and 12 h of light under humidity conditions of 55 ± 15%. The animals had free access to food and water. The experimental protocols were in accordance with the standards of the Chinese Ministry of Science and Technology for the Care and Use of Laboratory Animals after approval by the Animal Care and Experiment Review Board of Shanghai Traditional Chinese Medicine Hospital (Shanghai, China) (approval no. 20190103).

### 2.2. Establishment of the PCOS Rat Model and Treatments

The rats were divided into nine batches of 12 rats each: (1) the control group consisting of rats intragastrically administered with physiological saline; (2) the PCOS group consisting of PCOS rats with intragastric administration of physiological saline; (3) the PCOS+vehicle group containing of PCOS rats with administration of DMSO in physiological saline; (4) the PCOS+CRY group containing PCOS rats with daily intragastric administration of CRY; (5) the PCOS+ferrostatin-1 group containing PCOS rats with daily intragastric administration of saline and daily intraperitoneal administration of ferrostatin-1, the ferroptosis inhibitor; (6) the PCOS+CRY+erastin group containing PCOS rats with daily intragastric administration of CRY (27 mg/kg) and intraperitoneal administration of erastin; (7) the PCOS+MAPK inhibitor group containing all PCOS rats with daily intraperitoneal administration of 100 *μ*L Skepinone-L (10 mg/kg; China); and (8) the PCOS+CRY+Skepinone-L (selective p38*α*-MAPK inhibitor) group containing all PCOS rats with daily intraperitoneal administration of 100 *μ*L Skepinone-L (10 mg/kg; China). Ferrostatin-1 and erastin were dissolved in DMSO and diluted in physiological saline (0.9% NaCl).

The PCOS model was established as described in our previous study. Briefly, rats were administered by 2 daily subcutaneous injections with HCG (3.0 IU/day) and insulin for a duration of 22 days. The insulin dose was gradually increased from 0.5 to 3 U/day from days 1 to 11 and maintained at 3 U/day from days 12 to 22. Rats in the control group were treated with 2 skin injections of physiological saline. At the beginning of the experiment, water was replaced by 5% dextrose solution. Rats were weighed weekly, and vaginal swabs were taken daily from day 1 to day 23. Confirmation of PCOS was confirmed by the loss of regularity of the estrous cycle.

### 2.3. Assessment of Body Mass Index, Lee's Index, and Ovarian Quotient

At the end of the experiment, the length of the rats from the nose to the anus was measured and used to calculate Lee's index [42] and body mass index [43]. The formula for calculating Lee's index was as follows: Lee′s index = weight1/3 × 10^3^/length. The formula for calculating the body mass index was BMI = weight/length^2^. The unit of length was in centimeter while weight was in grams (g). Ovarian quotient was calculated as the quotient of ovarian mass to body mass and expressed in milligrams per 100 g.

### 2.4. Collection of Samples

At the end of the experiment, the rats were anaesthetized by intraperitoneal injection of sodium pentobarbital (55 mg/kg) after an overnight fast. Blood (5-7 mL) was collected from the abdominal aorta and subjected to centrifugation (4°C; 1,500 × g; 20 min) for serum collection. After this, pentobarbital sodium (250 mg/kg) was used to kill the animals and death was confirmed by exsanguination. Dissection of the ovaries was then performed, followed by weighing. For the immediate experiments, a part of the samples was fixed in a 4% paraformaldehyde solution at 25°C for 24 hours. The rest of the samples were stored in a refrigerator at -80°C.

### 2.5. Histopathological Analysis

For histomorphometric analysis, the tissues were successively dehydrated in graded concentrations of ethanol (50, 70, 80, 90, and 100%) for 30 sec. Afterwards, the tissues were washed in xylene and embedded in paraffin to make 4 *μ*m thick slices. The slices thus made were subjected to picric acid staining at room temperature for 30 min and hematoxylin-eosin staining at room temperature for 15 min. Finally, the stained sections were examined under a fluorescence microscope with the Leica DM5000 platform (Leica Microsystems, Inc.; magnification, ×100).

### 2.6. Immunohistochemistry

Protein expression was assessed by the immunohistochemical approach. Tissues were first fixed for 24 h in 4% paraformaldehyde at 4°C, embedded in paraffin, and cut into small 4 *μ*m thick slices. Subsequently, the tissues were blocked in 0.5% BSA solution followed by incubation with primary antibodies to GPX4 (1 : 200; cat. no. ab125066; Abcam), BAX (1 : 250; cat. no. ab32503; Abcam), NF-*κ*B (1 : 2000; cat. no. ab32536; Abcam), and HMGB1 (1 : 200; cat. no. Ab92310; Abcam) overnight. Revealing was done by visualization with biotin-conjugated secondary antibodies (1 : 300; cat. no. ab7176; Abcam) after half an hour incubation at 25°C using the Dako EnVision+ Detection System kit in strict accordance with the manufacturer's guidelines. Counterstaining of the coverslips was done by hematoxylin-eosin staining for 5 min at 25°C, and microscopic observation was done with the Leica DM5000 microscope (Leica Microsystems, Inc.; magnification, ×100).

### 2.7. Isolation and Culture of Rat Ovarian Granulosa Cells

Young female rats between 21 and 25 days of age were used to isolate granulosa cells from the ovary. The rats used in this study were commercially acquired from Shanghai Laboratory Animal Center, Co. Ltd. For this purpose, the rats were subjected to a subcutaneous injection of pregnant mare serum gonadotropin (PMSG) (150 IU/kg). 48 h after the injection, the rats were dissected and the ovaries were removed and subjected to follicular puncture as described above for the isolation of granulosa cells, after filtration and centrifugation for 5 min at 200 × g at 4°C. Subsequently, the supernatant was discarded and the cells were resuspended in Dulbecco's modified Eagles medium (Thermo Fisher Scientific, Inc.) to which compounds such as insulin, gentamicin, selenium, and transferrin were added. Cell culture was performed in 6-well plates at a density of 5 × 10^4^ cells/mL in an incubator set to a humidified atmosphere containing 5% CO_2_ for 24 h at 37°C.

### 2.8. Application of Ischemia-Reperfusion [28] to Granulosa Cells

Establishment of ischemia-reperfusion was done by treating granulosa cells with 1 *μ*mol/L dexamethasone for a period of 72 h, followed by determination of glucose and sucrose concentration with appropriate kits according to the vendor's recommendations.

### 2.9. Treatment and Determination of Cell Viability

Cells were subjected to different treatments including ischemia-reperfusion as described above, CRY, erastin, ferrostatin-1, and MAPK inhibitor. In other cases, several ferroptosis inhibitors were used. The treated cells were grown in 96-well plates at a density of 1 × 10^4^ cells per well. For the assessment of cell viability, the cells were treated with MTT reagent (0.2 mg/mL MTT) which was added to each well, followed by incubation in a humidified atmosphere containing 5% CO_2_ for 4 h at 37°C. Then, the formazan crystals were dissolved by treatment with DMSO and the absorbance at 490 nm was measured spectrophotometrically with microplate readers (Safire 2, Tecan Group, Ltd.).

### 2.10. Analysis of the Ultrastructure of Granulosa Cells

The ultrastructural changes of cells from different groups were analyzed using a transmission electron microscope. Briefly, GCs from different treatment groups were collected and after successive fixing in 2.5% glutaraldehyde and 1% phosphate-buffered osmium tetroxide, the GCs were embedded and colored using uranyl acetate and lead citrate. The transmission electron microscope (JEOL, Tokyo, Japan) was finally applied for microscopic imaging as well as analysis.

### 2.11. Intracellular ROS Measurement

The fluorescent 2′,7′-dichlorofluorescin diacetate probes (DCFH-DA) (Sigma-Aldrich, Poznan, Poland) were employed for the assessment of intracellular ROS. The GCs from different treatment groups were incubated in the dark with DCFH-DA (10 mM) at 37°C. Next, after rinsing three times, the cells were observed with the Olympus BX51 fluorescence microscope (Tokyo, Japan) for the detection of intracellular ROS fluorescence.

### 2.12. Terminal Deoxynucleotidyl Transferase dUTP Nick-End Labeling (TUNEL) Assay

A TUNEL-specific antibody was used for the histochemical staining of 6 *μ*m ovary sections. The sections were deparaffinized using Histo-Clear. Afterwards, following permeabilization in 0.3% Triton X-100, the DeadEnd™ Colorimetric TUNEL System (Promega, Madison, USA) was used for the detection of apoptosis in ovary tissues following the recommendations provided by the manufacturer. The Olympus IX81 microscope (Olympus America Inc., Center Valley, PA) was used for microscopic analysis, and green fluorescence was used for the identification of TUNEL-positive cells; counterstaining with the diamidino-2-phenylindole (DAPI) was used for the identification of nuclei.

### 2.13. RNA Extraction and RT-qPCR

RNA was extracted with the conventional method using the TRIzol extraction kit. The extracted RNA was retrotranscribed to cDNA using the GoScript™ Reverse Transcription System Kit (Promega Corporation) and following the protocols recorded therein. Amplification was done using the SYBR-Green PCR master mix platform supplied by Thermo Fisher Scientific, Inc. Thermal cycler settings were as follows: activation step at 50°C, denaturation at 95°C (30 seconds), 40 amplification cycles (95°C, 5 seconds), and termination (60°C, 30 seconds). The sequences of the primers used in the reaction mixture were recorded in Table 1.

### 2.14. Western Blot

For the western blot experiment, proteins were first extracted from the samples using RIPA reagent (cat. no. ab7937; Abcam). The protein-containing lysates were centrifuged and then subjected to quantification using BCA reagent (cat. no. 23227; Thermo Fisher Scientific, Inc.). Next, an aliquot of 50 *μ*g of protein was electrophoretically separated on 12% SDS-PAGE, followed by loading onto PVDF membranes and incubation in 25% skim milk for 120 min. The membranes were then contacted with solutions of primary antibodies directed against the indicated proteins. The antibodies used were PGC1a monoclonal antibody (1 : 5000, cat. no. 66369-1-Ig) from Proteintech, anti-NRF1 antibody (1 : 1000, cat. no. ab175932) from Abcam, GPX4 monoclonal antibody (1 : 1000, cat. no. 67763-1-Ig) from Proteintech, catalase monoclonal antibody (1 : 2000, cat. no. 66765-1-Ig) from Proteintech, ERK monoclonal antibody (1E5) (1 : 2000; MA5-15896) from Thermo Fisher, Phospho-p44/42 MAPK (Erk1/2) (Thr202/Tyr204) antibody #9101 (1 : 1000) from Cell Signaling Technology, anti-UCP2 antibody (1 : 1000, cat. no. sc-390189) from Santa Cruz, anti-Bax antibody (1 : 1000, cat. no. sc-7480) from Santa Cruz, BCL2 monoclonal antibody (1 : 2000, cat. no. 60178-1-Ig) from Proteintech, SOD1 monoclonal antibody (1 : 5000, cat. no. 67480-1-Ig) from Proteintech, Anti-NF-*κ*B p65 antibody [E379] (1 : 1000, ab32536) from Abcam, p38 MAPK (D13E1) XP® Rabbit mAb #8690 (1 : 1000) from Cell Signaling, and anti-beta Actin antibody (1 : 1000, ab8227) from Abcam. After incubation, the membranes were washed three times with TBST and incubated with the HRP-coupled secondary antibody solutions (1 : 5000; cat. no. ab7097; Abcam) at 25°C for 60 min. The revelation of the signals corresponding to the immune complexes was performed using the ECL reagent (cat. no. WBKLS0050; EMD Millipore). Finally, ImageJ software (Image J, National Institutes of Health, Bethesda, MD) was used for densitometric analysis of the bands. The ImageJ results were then used to calculate the relative expression of the proteins with reference to the Actin protein.

### 2.15. Immunofluorescence Staining

For protein (GPX4, BAX, NF-*κ*B, and HMGB1) expression in cells, GCs were subjected to immunofluorescence. GCs from different treatment groups were washed, and after fixing and incubation for blocking in 1% bovine serum albumin (BSA), GCs were incubated with primary antibodies (anti-GPX4, anti-BAX, anti-NF-*κ*B, and anti-HMGB1) at 4°C overnight. Then, the incubation with the secondary antibodies was performed in the dark for 1 h at 37°C. Finally, DAPI was used for counterstaining and examination under the Olympus BX51 fluorescence microscope.

### 2.16. Statistical Analysis

Data were expressed as mean ± sd. For comparison between two, the *T*-test was used. For analyses involving more than two groups, the one-way ANOVA test was performed; for comparative analyses between different groups, the Bonferroni post hoc test was applied following the one-way ANOVA. All analyses and graphs were produced with GraphPad Prism version 9 statistical software (GraphPad Software, Inc.).

## 3. Results

### 3.1. Ferroptosis Is Activated in Ovarian Granulosa Cells Subjected to Ischemia-Reperfusion

In order to investigate the probable involvement of ferroptosis in PCOS, we first treated granulosa cells with different ferroptosis inhibitors. The results showed that ferroptosis inhibitors had no cytotoxic effect on granulosa cells (Figure 1(a)). However, after ischemia-reperfusion, treatment of granulosa cells with the inhibitors showed different effects. Indeed, ischemia-reperfusion was followed by a remarkable decrease in cell viability (Figure 1(b)); but treatment with the different ferroptosis inhibitors was followed by a reversal of the effect of ischemia-reperfusion on cell viability. In addition, we found that the abrogation of the effect of ischemia-reperfusion was most pronounced after treatment with ferrostatin. Therefore, ferrostatin was selected as a ferroptosis inhibitor for further studies. These results indicated that ferroptosis activation may play a key role in the pathogenesis of PCOS.

### 3.2. CRY Inhibits Oxidative Stress by Regulating Ferroptosis via the MAKP Signaling Pathway

In order to elucidate the mechanism of action of CRY on the pathological processes involved in PCOS, we measured the effect of CRY on oxidative stress in the IR-induced PCOS model in vitro. The ultrastructural analysis indicated contracted mitochondria in the IR group and erastin groups while CRY and CRY+ferrostatin-1 treatment markedly improved the morphology of mitochondria (Figure 2(a)). In addition, the cotreatment of CRY with MAPK inhibitor or erastin significantly counteracted the effect of CRY on IR-induced cells (Figure 2(a)). The results also showed that IR and treatment with the ferroptosis stimulator, erastin, led to a decrease in cell viability (Figure 2(b)) and the activities of SOD (Figure 2(c)) and GSH-PX (Figure 2(d)). On the contrary, the level of MDA released in the PCOS model and in the erastin treatment group was increased compared to that in the control group (Figure 2(e)). Further study showed that ROS production was increased by PCOS or by erastin treatment (Figure 2(f)). In addition, we noted that treatment with CRY was followed by a reversal of the effects of erastin and PCOS on SOD, GSH-PX, MDA, and ROS (Figures 2(b)–2(f)). In addition, treatment with ferroptosis (ferrostatin) or MAPK inhibitor was followed by an effect similar to that of CRY. However, cotreatment with CRY and the ferroptosis activator (erastin) on the one hand and CRY and the MAPK inhibitor on the other was followed by a significant abrogation of the effect of CRY on PCOS. These results indicated that CRY inhibits PCOS-induced oxidative stress by regulating ferroptosis via the MAKP signaling pathway.

### 3.3. CRY Inhibits Mitochondrial Membrane Potential through Regulation of Ferroptosis via the MAKP Signaling Pathway

In order to detect whether CRY regulates oxidative stress through modulation of mitochondrial dynamics, JC-1 staining was performed. As shown in Figures 3(a) and 3(b), a significant decrease in red fluorescence was remarkable in the PCOS and erastin groups, leading to a drop in the ratio of red to green fluorescence, compared to the control group. In contrast, treatment with CRY alone or together with ferrostatin counteracted this effect. However, cotreatment of CRY with erastin or the treatment MAPK inhibitor reversed the effect of CRY on the ratio of red to green fluorescence. These results suggested that CRY inhibits mitochondrial membrane potential through the regulation of ferroptosis via the MAKP pathway.

### 3.4. CRY Inhibits GPX4 Expression and Activates NF-*κ*B via the MAKP Signaling Pathway in the PCOS Cell Model

In order to detect whether CRY regulates GPX4 and inflammation in the pathogenic processes of PCOS, immunofluorescence of GPX4 and NF-*κ*B was performed. As shown in Figures 4(a) and 4(b), a significant decrease in GPX4 expression was observed in the PCOS and erastin groups while NF-*κ*B expression was significantly increased in both groups compared to the control group. On the contrary, CRY and ferrostatin reversed the effect of erastin and IR-induced PCOS. However, cotreatment of CRY with erastin or the MAPK inhibitor inhibited the effect of CRY on GPX4 and NF-*κ*B expression levels. These results suggest that CRY inhibits PCOS-induced inflammation via the regulation of ferroptosis via the MAKP signaling pathway (Figure 4(c)).

### 3.5. CRY Inhibits HMGB1 and BAX Expression via Inhibition of Ferroptosis in the IR-Induced PCOS Cell Model

Immunofluorescence of HMGB1 and BAX was performed. As shown in Figures 5(a) and 5(b), significant activation of HMGB1 and BAX expression was observed in the IR and erastin groups. In contrast, CRY alone or in combination with ferrostatin abrogated the effect of erastin and IR on HMGB1 and BAX. However, cotreatment of CRY with erastin or the MAPK inhibitor inhibited the effect of CRY on HMGB1 and BAX expression levels (Figure 5(c)). These results suggest that CRY inhibits IR-induced HMGB1 and BAX expression via the regulation of ferroptosis.

### 3.6. Effect of CRY on Gene and Protein Expression In Vitro

In order to further confirm the mode of action of CRY, we determined the effect of CRY on the expression of genes involved in various biological processes associated with PCOS pathogenesis. At the transcriptional level (Figures 6(a)–6(e)), RT-PCR results showed that compared to the control group, IR treatment was followed by an inhibition of the expression of PGC1*α*, NRF1, GXP4, catalase, and SOD genes. Similar results were recorded with the ferroptosis activator, erastin (Figures 6(a)–6(e)). Furthermore, after treatment with CRY alone or in combination with the ferroptosis inhibitor (ferrostatin-1), the transcriptional levels of these genes increased compared to the IR group (Figure 6(a)), indicating an abrogation of the effect of IR and the ferroptosis inhibitor on these genes. In addition, treatment with the MAPK inhibitor abrogated the effect of cryptotanshinone, indicating an important role for MAPK in the mode of action of CRY (Figures 6(a)–6(e)). At the protein expression level, western blot results showed that the expression levels of PGC1*α*, NRF1, GXP4, catalase, SOD, p-ERK, UCP2, and Bcl2 were inhibited by treatment with IR and erastin but these inhibitory effects were reversed by treatment with cryptotanshinone alone or in combination with ferrostatin (Figure 6(f)). The effect of cryptotanshinone was also abrogated by treatment with the MAPK inhibitor (Figure 6(f)). A reverse trend was observed for Bax expression while no significant change was observed for ERK expression in the different groups (Figure 6(f)).

### 3.7. CRY Protects against the Deleterious Effects Underlying PCOS through Inhibition of Ferroptosis and Activation of MAPK

To verify the mode of action of CRY on PCOS in vivo, a rat model of PCOS was established. As shown in Figure 7(a), a regular structure of the rat ovary was observed in the control group, with numerous follicles (luteal, preantral, and antral) made of multiple layers with visible oocytes and corona radiata. In the PCOS and vehicle groups, microscopic examination showed cystic dilatation of the follicles with the presence of small layers of granulosa cells, the presence of corpora lutea, and lipid inclusions in the cytoplasm. However, treatment with CRY alone or with ferrostatin was followed by the presence of various follicles at different developmental stages and the presence of oocyte and corona in the mature follicles; corpora lutea growth and a regular layer of granulosa cells were also observed. The effect of CRY was abrogated by MAPK inhibitor.

In addition, we sought to verify the effect of cryptotanshinone and ferroptosis on cell apoptosis in vivo (Figures 7(b) and 7(c)). The TUNEL assay was used, and staining of ovarian tissue sections showed that in the PCOS model, cell apoptosis was increased compared to the control group. Treatments with vehicle led to similar results. However, treatments with CRY alone or in combination with ferrostatin led to a decrease in cell apoptosis. In addition, MAPK inhibitor increased the apoptosis rate in the PCOS model and reversed the effect of CRY on cell apoptosis.

In addition, the body weight (Figure 7(d)), ovarian weight (Figure 7(e)), and ovary quotiety (Figure 7(f)) were all increased in PCOS model but decreased by the treatment with CRY alone or in combination with ferrostatin. MAPK inhibitor reversed the effect of CRY on uterus body weight (Figure 7(d)), ovarian weight (Figure 7(e)), and ovary quotiety Figure 7(f). Moreover, hormonal tests indicated that Lee's index (Figure 7(g)) and BMI (Figure 7(h)) were all increased in the PCOS group but reversed by the treatment with CRY and CRY+ferrostatin-1; the effect of CRY was counteracted by the treatment with MAPK inhibitor. In addition, hormonal tests indicated that FSH (Figure 7(i)), LH (Figure 7(j)), and LH/FSH (Figure 7(k)) ratio as well as the testosterone (Figure 7(l)) levels were all increased in the PCOS group but reversed by the treatment with CRY and CRY+ferrostatin-1; however, treatment with the MAPK inhibitor counteracted the effect of CRY.

Immunohistochemistry was used to check the expression of proteins such as GPX4, BAX, NF-*κ*B, and HMGB1. As shown in Figures 8(a) and 8(b), in the PCOS group and after treatments with erastin and MAPK inhibitor, a decrease in the expression of GPX4, BAX, NF-*κ*B, and HMGB1 was observed in ovarian tissues whereas treatment with CRY and ferrostatin-1 was followed by an abrogation of this effect characterized by an increase in cells staining positive for these proteins. Moreover, the effect of CRY was counteracted by the treatment with the MAPK inhibitor (Figures 8(c) and 8(d)).

In order to further confirm the mode of action of CRY in vivo, we determined the effect of CRY on the expression of genes involved in various biological processes associated with the pathogenesis of PCOS. At the transcriptional level (Figures 9(a)–9(e)), RT-PCR results showed that compared to the control group, an inhibition of the expression of PGC1*α*, NRF1, GXP4, catalase, and SOD genes was observed in the PCOS group. Furthermore, after treatment with CRY or CRY+ferrostatin-1, the transcriptional levels of these genes increased compared to the PCOS group (Figures 9(a)–9(e)), indicating an abrogation of the effect of PCOS on these genes. In addition, treatment with the MAPK inhibitor abrogated the effect of CRY, indicating an important role for MAPK in the mode of action of CRY (Figures 9(a)–9(e)). At the protein expression level, western blot results showed that the expression levels of PGC1*α*, NRF1, GXP4, catalase, SOD, p-ERK, UCP2, and Bcl2 were inhibited by treatment with PCOS and erastin but these inhibitory effects were reversed by treatment with CRY or CRY+ferrostatin-1 (Figure 9(f)). The effect of CRY was also abrogated by treatment with the MAPK inhibitor (Figure 9(f)). A reverse trend was observed for Bax expression while no significant change was observed for ERK expression in the different groups (Figure 9(f)).

## 4. Discussion

Recent studies have demonstrated the crucial importance of ferroptosis in various biological processes such as cancers and cardiovascular and neurodegenerative diseases [33, 35, 44–47]. Studies have also shown that ferroptosis could affect the therapeutic efficacy of various drugs in the treatment of these diseases by promoting drug resistance [48–50]. In one of our previous studies, we proved the efficacy of CRY in the treatment and prevention of PCOS [28]. Other researchers have also reported the efficacy of CRY in the treatment of various ovarian conditions, including PCOS [24–27]. In addition, some undetailed studies by other investigators have suggested that ferroptosis may play an important role in the pathogenesis of PCOS [51, 52]. Thus, in the present study, we proposed to investigate the role of ferroptosis in the mechanisms underlying PCOS and to verify whether the mechanism of action of CRY could be mediated by its inhibitory action on ferroptosis. In this line, we conducted in vitro experiments by subjecting granulosa cells to ischemia-reperfusion and to treatments with CRY, inhibitors, and activators of ferroptosis and of the inhibitor of MAPK signaling pathway. Our results demonstrated in vitro and in vivo that ferroptosis was increased in cells subjected to IR in vitro and in the PCOS model in vivo. In addition, treatment with the ferroptosis activator and the MAPK inhibitor showed results with trends similar to the PCOS model. In contrast, treatments with CRY and the ferroptosis inhibitor were followed by a reversal of the effect observed in the PCOS model. In addition, the same trends were reported with respect to MMP, ROS, and expression of oxidative stress-related genes as well as apoptosis. These results indicate that the mechanism of action of CRY in the treatment of PCOS relies on its mediating effect on cellular ferroptosis. These results are of great value in the treatment and prevention of PCOS.

The results of the present study showed that ferroptosis levels were increased in granulosa cells subjected to IR and in the PCOS model in vivo. To date, specific studies investigating the role of ferroptosis in PCOS have not been reported. Only a few studies have reported the role of ferroptosis in ovarian cells or pathological conditions related to PCOS. An earlier study reported that uterine or placental ferroptosis can be modulated by insulin resistance and hyperandrogenism [51]. The sensitivity of clear cells found in the kidney and ovary to ferroptosis was also reported in another study which indicated that this sensitivity is based on the inhibition of GPX4 [52]. Proteomic analysis of CD4+ T cells from infertile PCOS patients showed that key proteins were involved in the ferroptosis pathway [50]. Differential gene expression analysis also demonstrated that crosstalk between autophagy, apoptosis, and ferroptosis is involved in the initiation of follicular atresia in pig ovaries [53]. Treatment of ovarian cells with the ferroptosis inhibitor reverses cellular cytotoxicity [54]. In view of the above, our study is the first of its kind to elucidate the involvement of ferroptosis in PCOS.

The effects of ferroptosis inhibitor and activator on MMP, ROS, and the expression of proteins involved in oxidative stress, inflammation, and apoptosis suggest that activation of ferroptosis in PCOS follows a deregulation of mitochondrial dynamics, promotion of inflammatory stimulation, and exacerbation of oxidative stress. These results corroborate those of a large body of literature showing an interconnection between ferroptosis and oxidative stress [55]. Furthermore, our results are consistent with other studies suggesting that oxidative stress is induced during the process of ferroptosis [56, 57]. Other studies have shown that during the regulation of ferroptosis, consequent changes occur at the mitochondrial level, including morphological changes, change in energy metabolism, change in iron metabolism, and change in lipid metabolism [58]; these results are in line with the results of the present study showing an effect of depolarization of MMPs by induction of ferroptosis. Our results are in line with those of other researchers also indicating that oxidative stress is induced by free radicals released during ferroptosis [59]. In this context, oxidative stress is induced by mitochondrial ROS release [59], which is consistent with the results of the present study showing the induction of ROS production by the activator of ferroptosis. However, the present study could only demonstrate the role of ferroptosis on oxidative stress and mitochondrial dynamics. Further studies are needed to confirm the directionality of the regulation between ferroptosis and oxidative stress as this outcome is equivocal. Indeed, although the studies cited above have confirmed the trend of our results, other researchers have shown that oxidative stress is a positive regulator of ferroptosis. For example, it has been reported that induction of oxidative stress by arsenite leads to induction of ferroptosis [60]. It has also been shown that oxidative stress induces ferroptosis and mitochondrial dysfunction in the retinal pigment cells PC12 [38, 61, 62].

CRY is known to have therapeutic and prophylactic benefits in a variety of diseases including ovarian, colon, bladder, and lung cancers and pulmonary fibrosis [12, 63–66]. CRY has also been reported to be effective against ovarian disorders, including PCOS [28, 67]. In many diseases, studies have demonstrated the mode of action of CRY by assessing its effect on a number of biological processes and signaling pathways. However, no study has evaluated the effect of CRY on disease-associated ferroptosis, especially in PCOS. Our present study therefore has the merit of demonstrating that CRY inhibits cell death by ferroptosis in PCOS. These results are of paramount importance as ferroptosis is considered a promising pharmacological therapeutic target for various diseases. Inflammation also plays an important role in PCOS. Many studies have shown a stimulation of inflammation in PCOS. In our previous study, we demonstrated that CRY inhibits inflammation by inhibiting metabolic pathways involving the NF-*κ*B protein. These results were confirmed in the present study. In addition, numerous studies have shown that ferroptosis involves inflammatory pathways involving the inflammasome. Although we did not measure the effect of CRY on the inflammasome, the regulation of NF-*κ*B by CRY is an indication that activated cellular ferroptosis in PCOS may be the result of an inflammasome activation cascade. Further study involving the NLRP3 inflammasome may clarify this hypothesis in our future studies.

We also noticed that CRY inhibits the MAPK/ERK pathway via inhibition of ferroptosis. Many studies have shown the connection between ferroptosis and the MAPK/ERK signaling pathway. According to the results of these studies, in case of ferroptosis, the MAPK/ERK pathway is activated. The activation of MAPK/ERK is also induced by the production of ROS in the medium. Here, we also noticed that HMGB1 protein was also upregulated in the PCOS model but inhibited by treatment with CRY and the ferroptosis inhibitor. Previous studies have shown a regulatory link between HMGB1 and the MAPK/ERK pathway. Therefore, we deduce that CRY exerts its therapeutic effect on PCOS by inhibiting the HMGB1/MAPK/ERK pathway via the induction of ferroptosis. There are still some limitations that remain to be solved in this study. Although CRY can decrease the expression of HMGB1 and NF-*κ*B in rats with PCOS, the underlying mechanism remains unclear. Besides, the protective effects of CRY on IR-induced ovarian granulosa cells were not confirmed through validation experiments other than cell viability detection. Still, cryptotanshinone may be a potential treatment option for polycystic ovary syndrome and the efficacy and safety of this mechanism need to be further studied.

## 5. Conclusions

In conclusion, the present study explored the mode of action of CRY on PCOS. The results demonstrate for the first time that ferroptosis is upregulated in PCOS and that the therapeutic or protective effect of CRY may be mediated by inhibition of this process which is a regulator of the HMGB1/MAPK/ERK pathway involved in the regulation of many pathological processes. This study provides a new perspective on understanding the pathogenesis of PCOS and offers hope in the search for therapeutic compounds for PCOS.

## Figures and Tables

**Figure 1:** Ferroptosis is activated in ischemia-reperfusion- (IR-) induced injury of granulosa cells. (a) Effect of different ferroptosis inhibitors on cell viability. (b) Effect of IR alone or in combination with ferroptosis inhibitors on cell viability. ns: nonsignificant. ^∗^*p* < 0.05, ^∗∗^*p* < 0.01, ^∗∗∗^*p* < 0.001, and ^∗∗∗∗^*p* < 0.0001, compared to control; ^#^*p* < 0.05 compared to IR.

**Figure 2:** Cryptotanshinone inhibits ischemia-reperfusion-induced oxidative stress by regulating ferroptosis via the MAKP signaling pathway in granulosa cells. (a) Ultrastructural analysis of GCs by transmission electron microscopy. (b) Effect of different treatments on cell viability. (c) Effect of different treatments on SOD. (d) Effect of different treatments on MDA. (e) Effect of different treatments on GSH-PX. (f) Effect of different treatments on ROS production. ns: nonsignificant. ^∗^*p* < 0.05, compared to control; ^#^*p* < 0.05 compared to IR; ^$^*p* < 0.05 compared to IR+CRY; ^&^*p* < 0.05 compared to IR+CRY+ferrostatin-1.

**Figure 3:** Cryptotanshinone regulates ischemia-reperfusion-induced mitochondrial membrane potential by regulating ferroptosis via the MAKP signaling pathway in granulosa cells. (a) Fluorescence image of GCs stained with JC-1 after different treatments. (b) Numerical data of green/red fluorescence-positive GCs. ^∗^*p* < 0.05, compared to control; ^#^*p* < 0.05 compared to IR; ^$^*p* < 0.05 compared to IR+CRY; ^&^*p* < 0.05 compared to IR+CRY+ferrostatin-1.

**Figure 4:** Immunofluorescence analysis of GPX4 and NF-*κ*B regulated by cryptotanshinone under ischemia-reperfusion injury. (a) Fluorescence image of GCs stained with GPX4 and NF-*κ*B after different treatments. The photograph shows GPX4 and NF-*κ*B and merge images. (b) Numerical data of the expression of GPX4-positive cells. (c) Numerical data of the expression of NF-*κ*B-positive cells. ^∗^*p* < 0.05, compared to control; ^#^*p* < 0.05 compared to IR; ^$^*p* < 0.05 compared to IR+CRY; ^&^*p* < 0.05 compared to IR+CRY+ferrostatin-1.

**Figure 5:** Immunofluorescence analysis of BAX and HMGB1 regulated by cryptotanshinone under ischemia-reperfusion injury. (a) Fluorescence image of GCs stained with BAX and HMGB1 after different treatments. The photograph shows MAPK and HMGB1 and merge images. (b) Numerical data of the expression of MAPK-positive cells. (c) Numerical data of the expression of HMGB1-positive cells. ^∗^*p* < 0.05, compared to control; ^#^*p* < 0.05 compared to IR; ^$^*p* < 0.05 compared to IR+CRY; ^&^*p* < 0.05 compared to IR+CRY+ferrostatin-1.

**Figure 6:** mRNA and protein expression regulated by cryptotanshinone under ischemia-reperfusion injury. (a) mRNA expression of PGC1a as determined by RT-qPCR. (b) mRNA expression of NRF1 as determined by RT-qPCR. (c) mRNA expression of GPX4 as determined by RT-qPCR. (d) mRNA expression of catalase gene as determined by RT-qPCR. (e) mRNA expression of SOD1 as determined by RT-qPCR. (f) Blot images and numeric quantification of protein expression of PGC1a, NRF1, GPX4, catalase, ERK, p-ERK, UCP2, BAX, and BCL2 as determined by western blotting. ^∗^*p* < 0.05, compared to control; ^#^*p* < 0.05 compared to IR; ^$^*p* < 0.05 compared to IR+CRY; ^&^*p* < 0.05 compared to IR+CRY+ferrostatin-1.

**Figure 7:** Cryptotanshinone protects against the deleterious effects underlying PCOS through inhibition of ferroptosis and activation of MAPK. (a) Histopathological analysis of ovary tissues obtained from different treatment groups. (b) TUNEL staining of ovary tissues obtained from different treatment groups. (c) Proportion of TUNEL-positive cells of ovary tissues obtained from different treatment groups. (d) Body weight or animals in different groups, (e) Ovarian weight from different groups. (f) Ovary quotiety in different groups. (g) Lee's index. (h) BMI of animals in different groups. (i) FSH level in different groups. (j) LH level in different groups. (k) LH/FSH ratio in different groups. (l) Testosterone level in different groups. ^∗^*p* < 0.05, compared to control; ^#^*p* < 0.05 compared to IR; ^$^*p* < 0.05 compared to IR+CRY; ^&^*p* < 0.05 compared to IR+CRY+ferrostatin-1.

**Figure 8:** Immunohistochemistry analysis of proteins. (a) Immunohistochemistry analysis of GPX4 protein of ovary tissues obtained from different treatment groups. (b) Immunohistochemistry analysis of BAX protein of ovary tissues obtained from different treatment groups. (c) Immunohistochemistry analysis of NF-*κ*B protein of ovary tissues obtained from different treatment groups. (d) Immunohistochemistry analysis of HMGB1 protein of ovary tissues obtained from different treatment groups.

**Figure 9:** mRNA and protein expression regulated by cryptotanshinone in PCOS. (a) mRNA expression of PGC1a as determined by RT-qPCR. (b) mRNA expression of NRF1 as determined by RT-qPCR. (c) mRNA expression of GPX4 as determined by RT-qPCR. (d) mRNA expression of catalase gene as determined by RT-qPCR. (e) mRNA expression of SOD1 as determined by RT-qPCR. (f) Blot images and numeric quantification of protein expression of PGC1a, NRF1, GPX4, catalase, ERK, p-ERK, UCP2, BAX, and BCL2 as determined by western blotting. ^∗^*p* < 0.05, compared to control; ^#^*p* < 0.05 compared to IR; ^$^*p* < 0.05 compared to IR+CRY; ^&^*p* < 0.05 compared to IR+CRY+ferrostatin-1.

**Table 1:** List of primers used in this study.

	Forward primer 5′→3′	Reverse primer 5′→3′
PGC1a	AGGTCCCCAGGCAGTAGAT	CGTGCTCATTGGCTTCATA
NRF1	TGGTGTCACTGGGCTCAATC	GTCTCAAGCTCTGGCCGAAT
GPX4	GGGGACAAAGAGCCGGTAG	GGTTACTGGGACCTAGGGGA
Catalase	CCACTCTCTCAGGAATCCGC	GGGTTCAGCTGTGCTGACT
ERK	CAGGCGCTGAGAGGAGAAAA	TGCTGCTAAGCCCATGGAAA
UCP2	CAATGTTGCCCGAAATGCCA	AGTTGGGTGAGGGGATCCAA
BAX	CTGAGACACTCGCTCAGCTT	TTGCTACAGGGGTGAGTGTG
BCL2	CCCCACAATGGTATGGCACT	CTGCAACACTGCTCTTTGCC
SOD1	AGCCCTATTGGTGAAGCAGA	TGTTTCCTTGCTCGTGGCTA
NF-*κ*B	CAACGCTGTCTCTCACTGGT	GACTGCCTTGACTTCCGTGA
MAPK	GGAGGGGCTCCTTTGAACTT	TGCTCCCTCTCATATCCCACA
Actin	AGGGAAATCGTGCGTGACAT	ACAACTACAGGGCTGACCAC

## Data Availability

All data generated or analyzed during this study are included in this published article.

## Abbreviations

PCOS: Polycystic ovary syndrome
CRY: Cryptotanshinone
ROS: Reactive oxygen species
IR: Ischemia-reperfusion
MMP: Mitochondrial membrane potential
LH: Luteinizing hormone
FSH: Follicle-stimulating hormone.
